# Application Research on Face Image Evaluation Algorithm of Deep Learning Mobile Terminal for Student Check-In Management

**DOI:** 10.1155/2022/3961910

**Published:** 2022-08-16

**Authors:** Yuanyuan Tan

**Affiliations:** School of Urban Geology and Engineering of Hebei University of Geosciences, Shijiazhuang 050031, Hebei, China

## Abstract

With the increase in the number of data, the traditional shallow image features cannot meet the needs of image representation. As an important means of image research, deep learning network has been paid attention to. In the field of face image evaluation, deep learning algorithm has been introduced, and the recognition technology has gradually matured. Based on this, this paper studies the application of face image evaluation algorithm of deep learning mobile terminal for student check-in management. A face image detection model for student check-in management is constructed, and a deep learning network is used to realize face detection. A face detection algorithm based on candidate region joint deep learning network is designed, and a face key point detection method based on cascaded convolution network is proposed. Aiming at the low efficiency of face recognition and detection, the existing loss function is optimized, the extraction algorithm of face binary features is proposed, and experiments are designed to analyze the performance of the algorithm. The simulation results show that the face detection based on the improved deep learning network can shorten the retrieval time and improve the accuracy of face image classification.

## 1. Introduction

Face detection refers to the process of determining the position and size of all faces (if any) in the input image. As a key technology in face information processing, face detection has become a popular and active research topic in the field of pattern recognition and computer vision. The original source of face detection and face recognition and the research on face recognition can be traced back to the 1960s and 1970s. After decades of tortuous development, it has become more and more mature. Face detection is a key part of automatic face recognition system, but early face recognition research mainly focused on face images with strong constraints, often assuming that the face location is known or easy to obtain, so face detection has not been paid enough attention to. In recent years, with the development of e-commerce and other applications, people have increasingly urgent requirements for automatic face recognition. Today, the application background of face detection has gone far beyond the scope of face recognition. It has important application value in artificial emotion computing, content-based retrieval, digital video processing, visual detection, and so on. With the progress and development of science and technology, colleges and universities began to use the new system to realize school management. In the field of student check-in, it has gone through many processes from previous artificial authentication to fingerprint scanning, infrared scanning, wireless RF scanning, and so on. These operation methods have their own advantages, but they also have their own defects [1, 2]. These check-in methods need professional equipment, the design and use cost are very high, and the operation is not convenient [3, 4]. With the popularity of smartphones, face image detection has been paid more attention to, and it is more suitable for sign-in management [5]. At present, face detection has made great progress, and technology has made some progress, but it is rarely applied to the field of university management.

The innovation of this paper lies in the retrieval algorithm of face recognition algorithm and neural network model training. Most feature extraction algorithms are based on high-dimensional Euclidean space, which is rich in information, but the retrieval time is long. This paper obtains binary features through the network, which effectively improves the efficiency of retrieval. In order to solve the problem of insufficient classification accuracy in the training and testing of binary classification convolution neural network, a method to improve the network structure is proposed. The dropout method is optimized, and the ReLU activation function is optimized. Combined with the regional recommendation method, the classification accuracy of network training is improved.

Based on this background, this paper studies the application of deep learning mobile face image evaluation algorithm for student check-in management, which is mainly divided into four sections. The first section briefly introduces the current situation of face recognition and detection for student management and the section arrangement of this research. Section 2 introduces the research on face image detection and deep learning algorithm and summarizes the shortcomings of the current research. In Section 3, a face detection system based on the mobile terminal of deep students is constructed, which is realized by using the deep learning algorithm. The face detection algorithm of candidate region generation volume and neural network classification is designed and compared with the traditional convolution learning network. Aiming at the problem of overfitting of face detection, the network structure is optimized, and the algorithm of region recommendation combined with convolution network is proposed. In Section 4, the deep learning mobile face image evaluation algorithm constructed in this paper is simulated and analyzed, and the running time, classification accuracy, detection accuracy, and other indicators are compared and analyzed. The results show that the improved ReLU function has the best convergence effect and the fastest convergence speed, and the classification accuracy of the improved dropout activation function network is 94.6%. After the improvement, the accuracy of network classification can be significantly improved. The accuracy of network classification under the improved algorithm shows great advantages. The candidate region recommendation algorithm has the highest face detection performance and can also shorten the detection time.

## 2. State of the Art

With the progress of computer technology, face detection has become one of the hot topics in the field of computer vision. Face detection is the basis of comprehensive recognition. It can quickly realize identity authentication from basic image acquisition to face detection, face location, face recognition, and other links [2, 6]. The research on face detection technology has also developed from the initial similarity detection to the current accurate location. For example, Luo and Guan proposed an adaptive skin detection method based on face location and face structure estimation in their research and analysis. The color spatial distribution model of facial skin is very close to that of real facial skin [7]. In their research, Zhou et al. combined a pair of near-infrared (NIR) cameras and a thermal camera (long wave infrared camera) and designed and prototyped a new hybrid sensor to capture the target and locate the 3D position of the eyes and face [8]. Gza and Yx. proposed an efficient face detection and tracking framework based on deep learning, including the SENResNet face detection model and face tracking (RNFT) model based on regression network. SENResNet model combines squeeze and excitation network (SEN) with residual neural network (RESNET) and uses RESNET to overcome the problem of gradient disappearance in deep neural network training [9]. Tao et al. proposed to use the Omega shape formed by human head and shoulder for head positioning in order to solve the problem of serious facial occlusion and constructed a new elliptical head contour detection energy function. The algorithm uses gradient and shape cable under the Bayesian framework [10]. Cho et al. proposed a two-step fast regional convolution neural network (R-CNN) based on histogram equalization (HE) preprocessing image, which successively executes the detectors of body and face regions and locates the face in a limited body region [11]. Duan et al. proposed a method to better represent the face detection image by feature fusion after deep convolution neural network (DCNN) feature extraction, reduce the dimension of fused features by PCA, and use support vector machine classifier to classify faces [12].

To sum up, we can see that there are many researches on face recognition and deep learning network. Most of the existing researches on face detection use task features for detection. The algorithms used are basically image geometric feature extraction, feature matching, or principal component analysis, which cannot deal with face recognition of complex images. Deep learning also has many algorithms in image target detection. The image is divided into multiple cells and grouped according to a certain level to find the similarity. This algorithm makes use of the transformation of classification problems and has a better detection effect. However, there are still many deficiencies in the application of deep learning algorithm, and it is rarely used in the field of university management. Therefore, it is of great practical significance to carry out the face detection system of deep student mobile terminal for student check-in.

## 3. Methodology

### 3.1. Portrait Detection for Student Check-In Management

In the era of big data, information technology is applied to university management. In the design of security system, the single-person management mode is no longer suitable, and the comprehensive management is based on scalability. Compared with other traditional recognition foundations, face detection technology has been paid attention to because of its good and concealment. In the system for student check-in, we should be able to accurately determine the identity of students and realize the online authentication of students' faces. According to the system requirements, face detection should cover two recognition bases. The first is face detection to ensure that the image is the image of students, and the second is face recognition to realize accurate analysis and sign-in of the image, as shown in Figure 1.

The performance and effect of face detection are closely related to the selection of core algorithms. The first is to perform smooth tracking based on some traditional tracking algorithms, such as the Kalman filter. The second is to directly predict the key points of video face based on the deep learning model. This directly affects the speed, accuracy, and stability of detection [13]. In face detection, the traditional VJ algorithm is based on integral graph feature extraction. It is relatively simple. Complex features will increase the computational complexity, resulting in slow detection speed and unable to meet the needs of student management. Face detection is a very complex detection problem, especially in the field of student check-in; it is also necessary to accurately recognize students' faces [14]. On the one hand, the face itself has many detailed changes, skin color is also an important influencing factor, and there are different expression characteristics. There will be some occlusion on the face, such as glasses and head ornaments. In the external conditions, the imaging angle will affect the face features, and the illumination factors and image imaging conditions will affect the detection results. Compared with traditional algorithms, the biggest function of deep learning algorithm is feature extraction. Compared with artificial design, the network can be regarded as a black box, which can directly obtain high-level features and simulate human cognition. It has strong adaptability in face detection. It is a commonly used feature extraction algorithm [15, 16].

### 3.2. Optimization Design of Deep Learning Algorithm

The deep learning network for face detection includes three layers: data layer, volume base layer, and red layer. It adopts a hierarchical overlapping link structure and intuitively adopts hierarchy. Each layer is formed by many neurons. In essence, it is considered that the detection adopts a binary classification network structure [17]. The convolution layer mainly calculates the image as a signal, and the formula is as follows:

(1) $$\begin{array}{c} X\left(x,y\right)*W\left(x,y\right)=\sum_{s=-w}^{w}\sum_{t=-h}^{h}W\left(s,t\right)X\left(x-s,y-t\right), \end{array}$$

where *X* represents the signal of the image and *W* represents the convolution kernel. In this calculation, every time the convolution kernel moves, the S matrix is obtained. Different convolution kernels are covered in the same layer, different features are output, and the features are input to the next layer network [18]. Pooling layer is a dimension reduction sampling process, which uses matrix to aggregate. When the maximum value is reached, the aggregation is expressed as follows:

(2) $$\begin{array}{c} x_{j}^{t}=f\left(\beta^{/}{\text{max}}_{i\in M_{j}}x_{i}^{t-1}+C^{/}\right). \end{array}$$

After multilayer network transmission, there will be great differences in the output results, which need to be normalized. The formula is as follows:

(3) $$\begin{array}{c} y=f\left(\sum w_{i}x_{i}+c\right), \end{array}$$

where *f* represents the activation function and the activation functions commonly used at present include Tanh, ReLU, and sigmoid functions. When the number of input data is, the probability distribution can be expressed as

(4) $$\begin{array}{c} p\left(y=i|x;\theta \right),\\ =\frac{e^{\theta_{i}^{T}x}}{\sum_{j=1}^{k}e^{\theta_{i}^{T}x}}, \end{array}$$

where *P* represents the probability and the label with the greatest probability is classification. Face detection belongs to nonlinear mapping, and the selection of classification function is very important for face detection. At present, the classification functions used are basically to select the data with great influence on the classification results and increase the weight [19]. Among many functions, the sigmoid classification function is suitable for multiclassification problems. This paper selects this classification function in classification. Sigmoid classification function transforms the output into probability distribution and then uses cross-entropy to replace the loss function. Through this function, the samples can be expressed as probabilities of different categories so as to predict the gap. However, in practical application, it is found that the gradient of the sigmoid function disappears, and the network cannot be effectively trained [20]. The formula of the ReLU function can be expressed as

(5) $$\begin{array}{c} f\left(x\right)=\left\{\begin{array}{cc} 0, & x\leq 0,\\ x, & x>0. \end{array}\right. \end{array}$$

When using this function, if the output value is greater than 0, it can ensure that the gradient will not disappear. However, when the output value of the ReLU function is less than 0, the network weight cannot be updated, so it needs to be improved. The formula is expressed as

(6) $$\begin{array}{c} f\left(x\right)=\left\{\begin{array}{cc} \alpha x, & x\leq 0,\\ x, & x>0, \end{array}\right. \end{array}$$

where *α* represents a parameter that can be learned. In face detection, the classification activation function of the initial network selects the improved ReLU activation function to accelerate the convergence and improve the detection accuracy. In face detection, the activation function is added at the volume base level, and all the following functions are changed to the ReLU activation function.

The change of light is the most important factor affecting the accuracy of face recognition. Because the face is a 3D structure, the shadow of light will enhance or weaken the original facial features. Secondly, the changes in facial expression can also affect the human face. Facial emotion change is composed of different small expression areas and finally face recognition acquisition angle. In face detection, overfitting is one of the main reasons for the low accuracy of face detection. When the model is overfitted, the classification cannot be carried out when new samples appear because there is more noise in the training set, resulting in insufficient adaptability of the model [21]. There are many image choices in face detection, and the problem of detection ability will appear when the details or noise are received in the learning of sample data. When solving the overfitting problem, it is generally to expand the dataset or regularize. In the iterative process, the program operation is ended in advance, and the method of ending the training in advance cannot determine the best end time. Theoretically, the more data, the better the training result. However, if the input data is too large, the data selected in the iteration may also be fitted. Adding a regular term after the loss function to improve the function structure is also one of the methods. Dropout does not change the input and output in application and randomly discards neurons according to a certain proportion. This improved method combines different coefficient models, randomly selects other neurons to write together, reduces the joint adaptability, avoids the phenomenon of network overfitting, and can also shorten the running time. At present, the common expression of dropout neural network is

(7) $$\begin{array}{c} z_{i}^{\left(l+1\right)}=w_{i}^{\left(l+1\right)}\overset{∼\left(t\right)}{y}+b_{i}^{\left(l+1\right)}. \end{array}$$

After the dropout function is added, the Bernoulli random distribution function is used to determine the neuron connection of the front and rear layers. Due to the randomness, the training structure will show diversity every time, which needs to be improved. The dropout method reduces the overfitting phenomenon through the random combination network of neural nodes at different levels, which will affect the final classification results. In network training, the network weight parameters will be continuously adjusted. In selective training, most of the values will be input into the connected node parameters, which will affect the training results. Dropout is encapsulated in the form of hierarchy. It needs to contact the full connection layer and neural nodes. The output and input of neural nodes have the following relationship:

(8) $$\begin{array}{c} y_{i}=\text{softmax}\left(x_{i}\right),\\ =\frac{e^{x_{i}}}{\sum_{i=l}^{n}e^{x_{i}}}, \end{array}$$

where *x* represents the output of the full connection layer and *y* represents the probability that the output is classified. When the output value is greater than half, it belongs to *i* class. *x* value is output when it can be clearly classified. The input increases exponentially, so the output changes greatly, and the classification results are more clear. In the training results, you can selectively train and let the larger value as the input parameter, and the others do not participate in the output. Specifically, the nodes input from the full connection layer are sorted. The data with small sorting is directly set to zero, and the nodes are not connected, so the larger results are output. The network architecture of this method contains multiple alternating pooling layers and convolution layers to form the basic image information and then extract the features. This algorithm adopts the strategy of joint traffic training, and only the basic eigenvectors are different.

### 3.3. Face Recognition

After determining that the input information is face information, continue face recognition, extract high-dimensional features, and judge the similarity according to Euclidean distance. However, this traditional method is inefficient, so it needs to be improved [22]. In this paper, the binary feature algorithm is used in face recognition. In order to distinguish different faces and get better feature information, we choose the deep network model of Google company, take Inception-ResNet-v2 as the core structure, and select the representative loss function for analysis and improvement. Residual network is a popular network model structure at present, so this paper selects this network model [4]. Compared with the convolutional neural network, the residual network has more bypasses, which can ensure the integrity of information. With the increase of network maturity, the residual network will not have the problem of degradation but also reduce the time complexity.

Sigmoid layer is the activation function in the deep learning network, similar to the synapse of neurons. In this paper, in face recognition, the function is not the activation function but maps the eigenvalue to the interval class of 0∼1 and binarizes the threshold [9]. The classification layer is connected with the sigmoid layer. Each individual corresponds to a category. The spacing is expanded through classification training. This function is classified through normalization. The formula is

(9) $$\begin{array}{c} y_{i}=\frac{e^{a_{i}}}{\sum_{k=1}^{c}e^{a_{i}}}\;\forall i\in 1.c. \end{array}$$

The introduction of softmax function can solve the gradient disappearance problem to a certain extent. Sigmoid function is suitable for the derivation of the cross-entropy loss function, which can be expressed as

(10) $$\begin{array}{c} c=-\frac{1}{n}\sum \left[y\;\ln\;a+\left(1-y\right)\ln\left(1-a\right)\right], \end{array}$$

where *a* represents the actual output result of the network and *y* represents the expected output result. By deriving *w* and *b*, we get

(11) $$\begin{array}{c} \frac{\partial c}{\partial w_{j}}=\frac{1}{n}\underset{x}{\sum }x_{j}\left(\delta \left(z\right)-y\right),\\ \frac{\partial c}{\partial b}=\frac{1}{n}\sum_{x}\left(\delta \left(z\right)-y\right). \end{array}$$

The derivation function can avoid the problem of gradient elimination in the sigmoid function. In the softmax classification layer, the purpose is to expand the distance between classes. The center distance loss layer can reduce the distance within classes. The formula is expressed as

(12) $$\begin{array}{c} C=\frac{1}{2}\sum_{i=1}^{m}{\left\|x_{i}-c_{y_{i}}\right\|}^{2}, \end{array}$$

where *c* represents the characteristic center value of the sample and *x* represents the characteristic value of the individual. Calculating the distance from each class sample to the class center as the loss value can reduce the variance between classes [23]. The loss between classes refers to the ternary loss of FaceNet and maintains the distance between classes. The formula is expressed as

(13) $$\begin{array}{c} y=\sum_{i}^{N}\left[{\left\|x_{i}^{a}-x_{i}^{p}\right\|}_{2}^{2}-{\left\|x_{i}^{a}-x_{i}^{n}\right\|}_{2}^{2}+a\right]. \end{array}$$

In the formula, *a* is the fixed threshold. This function is further simplified and expressed as

(14) $$\begin{array}{c} y=\sum_{i}^{N}\text{max}\left\{a-{\left\|x_{i}^{a}-x_{i}^{n}\right\|}_{2}^{2},0\right\}. \end{array}$$

It can be seen from the network layer that the whole deep learning network maintains the distance while maintaining the proximity of similar feature individuals. The sigmoid layer controls the mapping to 0∼1 and realizes feature binarization through threshold segmentation.

In the location and recognition of face key points, the information involved mainly covers the eyes, nose, and corners of the mouth, in which glasses are the geometric center. Among various network models, *F*1 model is the most widely used one with a simple structure, which is composed of multiple convolution layers, sampling layers, and connection layers. *F*1 network model requires good image quality and is easy to extract more feature information in face key point location and recognition. There is no nonlinear transformation in the application, and the network needs to add a nonlinear layer [24]. The *F*1 model needs to be improved. Increase the input face size information, increase the convolution kernel, and add the ReLU layer between the volume base layer and the first full connection layer to improve the performance of the network model.

When constructing the network structure, the three-level structure is adopted. Considering the high requirements of video detection speed, a certain simplification is carried out. The first level network is a full convolution network, which finds the face area. The number of convolution cores is set to 6, 10, 14, 2, and 4. This network structure is the most concise. The second level network has accurate positioning, the resolution of the input picture is 24^*∗*^24, and the number of convolution cores is more. The third level is the final recognition. The input resolution is 48^*∗*^48, and the number of volume base layers is four. The three-level network forms the model structure of the final candidate box, and the three-level network is tested after completion. The training set selects the public WIDER FACE benchmark dataset, which covers the faces with different occlusions and angle changes. The parallel cross ratio is used to determine the coincidence rate. Those higher than 0.65 are positive samples, and others are negative samples. Firstly, cut the pictures to 12*∗*12, and classify the samples according to the parallel cross-ratio. After the first level network is trained, it is used as the sample generator of the second level to obtain the candidate region. Each level of network has two classification layers, which are trained by the cross-entropy loss function.

## 4. Result Analysis and Discussion

### 4.1. Simulation Analysis of Loss Rate of Activation Function Classification

The model studies the application of the method in operational risk in detail. According to the quantitative methods and strategies of operational risk, this paper will establish a quantitative model of operational risk from the types of loss events, business departments, and the amount of loss distribution. At the same time, the definition of operational risk at risk is introduced to calculate the capital allocation of different risks. The performance of several activation functions is measured, and the changes in the classification loss rate of the sigmoid function, improved ReLU function, Tanh function, and PReLU function are compared.

Figure 2 shows the network classification results under different activation functions. As can be seen from Figure 2, the network classification is affected by the activation function. The sigmoid function has no obvious effect and no convergence. The improved ReLU function has the best convergence effect and the fastest convergence speed. Under the traditional activation function, it needs tens of thousands of iterations to converge, and the improved function can greatly reduce the number of iterations.

In the process of zeroing, array selection is very important. Select arrays with different zeroing rates for network training, and analyze the training results, as shown in Figure 3.

It can be seen from the data in the figure that when the zero setting rate is 0, it is a traditional deep learning network. When the zero setting rate is 10%, the early oscillation is intense, the convergence speed is full, and the accuracy is not very high. At this time, almost all neurons participate in it, there are many parameters, the convergence speed is slow, they are affected by the classification function, and the accuracy of the output result is not high. When the zero setting rate is 0.3 and 0.4, there is no great fluctuation in the early stage, the convergence speed is accelerated, the accuracy is also improved, and the performance is better when the zero setting rate is 0.4. Therefore, the network zero setting rate designed in this paper is 0.4.

The network training is carried out under the improved dropout method, which is improved on the basis of the original convolutional neural network. After the neural network is obtained, complete the file definition in prototype XT during the training. Set the network parameters with prototype text in solver, and use 64 memory pictures and 100000 maximum iterations. The GPU mode is used for training. The benchmark learning rate is 0.001, the momentum setting is 0.9, and the weight attenuation is 0.005. The parameters are initialized, tested with ImageNet dataset and self-built dataset, trained for 10 times, and compared and analyzed the network classification accuracy before and after the improvement. The classification accuracy of the original network model is 70.2%, that of the PReLU activation function is 89.3%, and that of the dropout activation function is 94.6%. After the improvement, the accuracy of network classification can be significantly improved. Further analyze the classification accuracy when the network converges under different algorithms. The measurement results are shown in Figure 4. From the figure, it can be seen that the network classification accuracy under the improved algorithm shows great advantages, and the classification accuracy has been significantly improved.

In the simulation analysis of face detection effect, there are two evaluation indexes that can be referred to: the overlap degree and detection time between the candidate region and the actual face region. When the overlap rate is 1, they are considered to be completely overlapped. The running time of the traditional algorithm is 1.4 s, the running time of the sliding window improved algorithm is 0.98 s, and the running time of the candidate region recommendation improved algorithm proposed in this paper is 0.23 s. The running time of the region recommendation improved algorithm proposed in this paper is significantly shorter than that of the other two algorithms. The detection overlap rate results are shown in Figure 5. It can be seen from the figure that the detection overlap rate of the improved algorithm in this paper is significantly higher than that of the other two algorithms, indicating that the candidate region recommendation algorithm proposed in this paper has the highest face detection performance and can also shorten the detection time.

The improved algorithm is used to detect the face of the image. The detection results are shown in Figure 6. It can be seen from the figure that, under different occlusion, angle, overlap, and other modes, all the improved algorithms proposed in this paper can be detected, and the detection results are ideal.

### 4.2. Face Recognition Simulation Analysis

In face recognition, for the image to be detected, select the minimum size to be detected, and then carry out size transformation. The first level network is a full convolution network. Input 12*∗*12 images to obtain the candidate box. Filter the repeated area by using the nonmaximum algorithm, and input the result into the second level network. The second level input picture size is 24*∗*24, and the third level input picture size is 48*∗*48. First, use the FDDB database for face detection. This database is the current authoritative face detection test platform, covering pictures with different postures, resolutions, and angles to test the accuracy of face recognition. The measurement results are shown in Figure 7. It can be seen from the figure that, under the simplified network structure, the accuracy of face recognition of the improved algorithm proposed in this paper is still relatively high.

Then test the face recognition effect in the video. Normally shoot the students' face pictures with a resolution of more than 20*∗*20. You can shoot with light and angle changes. Collect daily videos of students, covering undetected faces, a small number of faces, and face images of other students. The background is complex, and there are difficult factors such as lighting factors and angle changes. Detect each frame of image, save the detection results, adjust and classify the images with reference to the detection effect picture, and calibrate the database manually in real time. Test according to the calibrated picture, and test the sample with reference to the identification index. The average detection time of the traditional algorithm is 687 ms, and the average detection time of the improved algorithm is 620 ms, which significantly shortens the detection time of the algorithm. The accuracy of video face detection under different algorithms is shown in Figure 8. As can be seen from the figure, the detection accuracy of the proposed algorithm is improved compared with the traditional algorithm.

In the face feature point location test, the test set selects the internal set, detects the five feature points of the face, and measures the error rate. The measurement results are shown in Figure 9. It can be seen from the figure that no matter what model, the detection error rate of mouth corner is the highest, which may be because the change range of mouth corner is relatively large, so the error rate is high. Under the improved *F*1 model, the average prediction error rate of face detection has decreased significantly, especially the detection error rate of both eyes.

## 5. Conclusion

This paper studies the application of deep learning mobile terminal face image evaluation algorithm in student registration management. Aiming at the problem that the classification accuracy of the original deep learning network is not high, the activation function and network structure are improved. In order to improve the accuracy and efficiency of retrieval, a deep convolution network with the PReLU function as the activation function is proposed to extract binary features. The simulation results show that the face detection and classification accuracy of the improved deep learning network has been significantly improved, which proves the superiority of the algorithm. It should be pointed out that face detection in this paper considers the detection, recognition, and location of key points, which improves the retrieval speed. In this paper, binary features are obtained through the network, which effectively improves retrieval efficiency. Aiming at the problem of insufficient classification accuracy in training and testing of binary classification convolution neural network, a method to improve the network structure is proposed. The exit method and ReLU activation function are optimized. Combined with the regional recommendation method, the classification accuracy of network training is improved.

However, the study did not consider the problem of face alignment. There are great differences in different environments after binary feature extraction. We also need to consider how to reduce the difference in the individual distance through the training network.

## Figures and Tables

**Figure 1:** Face detection based on sign-in management.

**Figure 2:** Network classification under different activation functions.

**Figure 3:** Comparison of network classification accuracy of improved dropout method.

**Figure 4:** The correct rate of network classification before and after improvement.

**Figure 5:** Analysis of detection overlap rate.

**Figure 6:** Face detection effect.

**Figure 7:** Accuracy analysis of face recognition.

**Figure 8:** Monitoring results of video face detection accuracy under different algorithms.

**Figure 9:** Prediction error rate analysis under different models.

## Data Availability

The data used to support the findings of this study are included within the article.
